The article "Online Education Classroom Intelligent Management System Based on Tensor CS Reconstruction Model" was published in 2022. Journal: Comput Intell Neurosci.

# Online Education Classroom Intelligent Management System Based on Tensor CS Reconstruction Model

**DOI:** 10.1155/2022/9907786

**Published:** 2022-06-28

**Authors:** Hui Mu, Yali Shi

**Affiliations:** Department of Foundational Disciplines, Shijiazhuang People's Medical College, Shijiazhuang, Hebei, China

## Abstract

To study a high-efficiency online classroom intelligent management system, this article builds an artificial intelligence classroom management system based on the tensor CS reconstruction model. Moreover, this study uses the cosine function to represent the data energy fitting of the traditional active contour model and proposes a local cosine fitting energy active contour model based on partial image restoration, which is used for image and composite image segmentation. Simultaneously, this study proposes a new type of super-resolution algorithm. This algorithm performs Fourier transform of a low-resolution image into a frequency range and then performs an inverse Fourier transform on the image expanded in the frequency range to obtain the initial high-resolution image and finally reconstructs a new super-resolution image using the frequency-domain compressed data of the high-resolution image. Finally, this study verifies and analyzes the performance of the model through experiments. The research results are basically consistent with the expectations of the model.

## 1. Introduction

Smart teaching is the inevitable trend of future education. There is a certain difference between the classroom management of smart teaching and traditional classroom management, and the corresponding teaching system needs to be combined with the smart classroom teaching mode. Based on this, this article builds an online classroom intelligent teaching management system based on machine learning algorithms [1].

The difference between the traditional classroom and the smart classroom is that the smart classroom makes the traditional classroom more “smart” [2]. That is, a smart classroom can intelligently perceive situational information such as the classroom, students, and environment through related equipment and can make corresponding “actions” by judging and processing the feedback situational information, such as various reminders to students, online questions from students, teachers' timely feedback on students' questions, and recommendations to students that are equivalent to their learning level [3]. Regardless of whether it is a smart classroom or a traditional classroom, the classroom is used as a place for students to attend classes, as well as a place for students and teachers to exchange knowledge and academics with each other. With the differences in the location and learning status of students, classroom situation information can be roughly divided into the following parts: classroom location situation information, classroom time situation information, classroom environment situation information, student situation information, and classroom equipment situation information [4].

The article "Online Education Classroom Intelligent Management System Based on Tensor CS Reconstruction Model" was published in 2022. Journal: Comput Intell Neurosci.

With the popularization of computers and networks, my country's online education has also been fully developed, and many universities in our country have successively opened online education classes, providing a sufficient foundation for the development of distance online teaching. At the same time, major colleges and universities have begun to develop some teaching software that suits the characteristics of their colleges and universities, which has also accelerated the development of online education to a certain extent [5].

The network teaching platform is the concrete manifestation of modern informatization in teaching. In fact, it is a kind of teaching environment. It includes not only various computer equipment and multimedia equipment in hardware but also teaching software and operating system in software application [6]. The purpose is to assist in daily teaching. The content that it contains mainly includes course introduction and inquiry, teaching arrangement, and announcement. Moreover, it is a comprehensive teaching system that can achieve multiple functions. Nowadays, various industries have related online teaching platforms, including schools, hospitals, and enterprises. Moreover, with the development of technology, these teaching platforms are constantly updated and upgraded, and they have achieved considerable development in terms of function and performance.

## 2. Related Work

Low-rank models have richer mathematical properties than sparse models. In high-dimensional data, the rank of a matrix indicates the number of nonzero singular values of the matrix, and low rank means that fewer vectors can be used to represent the structure of the matrix. The literature proposed a low-rank representation-based subspace clustering algorithm (LRR) [7]. This model considers the joint multi-subspace clustering problem, divides the sample data into corresponding representative subspaces, and combines subspace segmentation and noise recognition in a framework. Sparse representation SR and low-rank representation LRR are the two most important ways of matrix representation. In data mining, SR is often combined with clustering. LRR can not only be used for clustering but also commonly used in matrix recovery applications [8]. At present, sparse and low-rank subspace clustering algorithms have been extensively studied. There are dozens of subspace clustering algorithms based on sparse and low-rank representations. On the basis of SSC, the literature extended the a priori condition of subspace independence to subspace disjointness and proposed a sparse subspace segmentation algorithm [9]. The literature required the coefficient matrix to be sparse while satisfying the positive definite condition and proposed a quadratic programming subspace division algorithm (SSQP) [10].

The article "Online Education Classroom Intelligent Management System Based on Tensor CS Reconstruction Model" was published in 2022. Journal: Comput Intell Neurosci.

According to the development process of feature selection algorithms, the current development of feature selection algorithms tends to be the combination of feature correlation and multiple algorithms. The more classic cluster-based feature selection algorithms are as follows. The literature proposed the multi-cluster feature selection method (MCFS). This method uses all the input features to represent the data structure, then embeds high-dimensional data into low-dimensional space through sparse features, sorts the features according to the regression method, and selects features that are easy to maintain the local popular structure [11]. Literature proposed an unsupervised discriminative feature selection (UDFS) method to make a partial judgment on each sample and obtain the feature subset with the highest score by solving the normalization problem [12]. However, when expressing the relationship between data, this method uses the distance function between samples, and once the function parameters are determined, all relationships use the same function, which does not conform to the law of data distribution. To solve this problem, a local learning clustering feature selection method (LLCFS) is proposed, which introduces correlation features into a regularized local learning model to enable the model to be optimized iteratively [13]. However, this method actually optimizes the two objective functions of structure learning and feature selection, and its theoretical convergence and practical results are not good. Most of the existing unsupervised feature selection methods cannot accurately estimate the data structure. On the one hand, the real structure of the data is required for feature recognition, and on the other hand, the feature is required to accurately estimate the real data structure. Based on this, an adaptive learning feature selection method is proposed. This method first extracts the global and local structure of the data, then obtains relevant features through unsupervised feature learning, and finally builds a sparse map through the obtained relevant features [14]. The adaptive learning feature selection method algorithm integrates structural features and unsupervised learning into the same framework. It is a feature selection algorithm that can be improved adaptively according to the data structure [15].

The article "Online Education Classroom Intelligent Management System Based on Tensor CS Reconstruction Model" was published in 2022. Journal: Comput Intell Neurosci.

## 3. Construction of Adaptive Learning Dictionary

The *i*th noise-containing image block *u*_*i*_ in the monitored image *Y* with an assumed size of $\sqrt{n}\times \sqrt{n}$ is considered, and *u*_*i*_ is arranged into a column vector *y*_*i*_ ∈ *R*^*n*^. To establish a sparse model, it is necessary to construct an over-complete dictionary *D* ∈ *R*^*n*×*k*^; among them, there is *k* ≫ *n*. For image *Y*, the sparse representation coefficient *α*_*ij*_ of dictionary *D* is obtained by the following formula:

(1) $$\begin{array}{c} \left\{{\hat{\alpha }}_{ij},\hat{X}\right\}=\arg\underset{\alpha_{ij},X}{\min}\lambda {\left\|X-Y\right\|}_{2}^{2}+\sum_{i,j}\mu_{ij}{\left\|\alpha_{ij}\right\|}_{0}+\sum_{i,j}{\left\|D\alpha_{ij}-R_{ij}X\right\|}_{2}^{2}. \end{array}$$

Among them, *i* and *j* are the data row and column directions, respectively; that is, the image block is located at the (*i*, *j*) position. The first item on the right is the similarity between the noise image *Y* and the denoised image *X*. Among them, *λ* is a parameter that controls the degree of punishment of the regularization item. The second term is the sparse constraint, where *μ*_*ij*_ is the penalty factor. In the third item, *R*_*ij*_ is a cropping operator used to extract small image blocks at pixel (*i*, *j*), and *R*_*ij*_*X* is a calculation formula for extracting and converting small image blocks into column vectors. *Dα*_*ij*_ is the small image block reconstructed by the column vector corresponding to the small image block *R*_*ij*_*X*, and the difference between *Dα*_*ij*_ and *R*_*ij*_ is as small as possible.

### 3.1. Solving Sparse Model

We assume that the dictionary *D* in the above formula is known, and the two unknowns of the output image *X* and the sparse coefficient ${\hat{\alpha }}_{ij}$ cannot be calculated at the same time. Therefore, to solve the equations of ${\hat{\alpha }}_{ij}$ and $\hat{X}$, we need to initialize *X*=*Y* first and then find the optimal coefficient ${\hat{\alpha }}_{ij}$:

(2) $$\begin{array}{c} {\hat{\alpha }}_{ij}=\arg\underset{\alpha_{ij}}{\min}\mu_{ij}{\left\|\alpha_{ij}\right\|}_{0}+{\left\|D\alpha_{ij}-R_{ij}x\right\|}_{2}^{2}. \end{array}$$

In the above formula, the coefficient column vector ${\hat{\alpha }}_{ij}$ of *R*_*ij*_*x* is calculated by selecting the value of *μ*_*ij*_. Once ${\hat{\alpha }}_{ij}$ is obtained, *X* is updated to the following form:

(3) $$\begin{array}{c} \hat{X}=\arg\underset{X}{\min}\left\{\lambda {\left\|X-Y\right\|}_{2}^{2}+\sum_{i,j}{\left\|D{\hat{\alpha }}_{ij}-R_{ij}X\right\|}_{2}^{2}\right\}. \end{array}$$

The above formula is a simple quadratic equation, and its closed solution has the following form:

(4) $$\begin{array}{c} \hat{X}={\left(\lambda I+\sum_{i,j}R_{ij}^{T}R_{ij}\right)}^{-1}\left(\lambda Y+\sum_{i,j}R_{ij}^{T}D{\hat{\alpha }}_{ij}\right). \end{array}$$

Among them, *I* is the identity matrix.

The article "Online Education Classroom Intelligent Management System Based on Tensor CS Reconstruction Model" was published in 2022. Journal: Comput Intell Neurosci.

### 3.2. Dictionary Learning

Once the dictionary *D* is known, the orthogonal matching pursuit (OMP) algorithm can be used to solve equation (2) to estimate the optimized coefficient matrix {*α*}_*j*=1_^*M*^. Moreover, the dictionary *D* can be adjusted according to the different characteristics of the band images that may contain noise.

To build a dictionary, formula (1) is redefined as follows:

(5) $$\begin{array}{c} \left\{\hat{D},{\hat{\alpha }}_{ij},\hat{X}\right\}=\arg\underset{D,\alpha_{ij},X}{\min}\lambda {\left\|X-Y\right\|}_{2}^{2}+\\ \sum_{i,j}\mu_{ij}{\left\|\alpha_{ij}\right\|}_{0}+\sum_{i,j}{\left\|D\alpha_{ij}-R_{ij}X\right\|}_{2}^{2}. \end{array}$$

First, the dictionary *D* and the image *X* to be denoised are initialized. Then, the OMP algorithm is used to estimate the sparse representation coefficient ${\hat{\alpha }}_{ij}$, as shown in formula (2). Secondly, on the basis of the estimated coefficient ${\hat{\alpha }}_{ij}$ and the initial denoising image *X*, the dictionary $\hat{D}$ in the above formula is updated using the K-SVD algorithm. Finally, formula (4) is used to update the denoised image $\hat{X}$.

All visible light and near-infrared bands of 13 Landsat − 7ETM+SLC − ON images are used, and the K − SVD algorithm is used for redundant dictionary training. To save space, each band selects only 5 of the 13 images to be displayed. In Figure 1, from left to right, the first to fifth columns correspond to the Flathead Lake area of Montana, USA, 08/03/1999, 09/20/1999, 10/08/2000, and 07/07/ ETM+ image obtained on October 14, 2002 and 2001. For each column, the rows from top to bottom correspond to bands 1, 2, 3, 4, 5, and 7, respectively. In the last column, 6 dictionaries corresponding to the 6 bands of the Landsat − 7 image obtained after training are displayed.

## 4. Image Restoration Model Based on Sparse Representation

To use the observed image *y* ∈ *ℂ*^*M*^ to repair the missing data, the image pixel missing model can be expressed as follows:

(6) $$\begin{array}{c} y=\Phi x. \end{array}$$

Among them, Φ ∈ *ℂ*^*M*×*N*^ is the missing operator, *x* is the image without any data loss or repaired image, and *y* is the observed data missing image. The missing pixel data are effectively estimated using the nonlocal information and global information of the Landsat − 7ETM+SLC − ON image. At the same time, a mathematical model is established through the relationship between the image *y* to be repaired and the image *x* after the repair. The sparse model based on image restoration can be expressed in the following form:

(7) $$\begin{array}{c} y=\Phi x+\varepsilon . \end{array}$$

Among them, *ε* is additive noise. For the over-complete word, *D*={*d*_1_, *d*_2_,…, *d*_*i*_,…, *d*_*M*_} dictionary, where *d*_*i*_ ∈ *ℂ*^*N*^ is the atom of the dictionary. If there is *M* ≫ *N*, *D* is called a redundant dictionary. To repair the image, the dictionary *D* can be sparsely decomposed into the following form.

The article "Online Education Classroom Intelligent Management System Based on Tensor CS Reconstruction Model" was published in 2022. Journal: Comput Intell Neurosci.

The 6 dictionaries are for Landsat − 7ETM + SLC − ON image training, and the training area is Landsat − 7ETM + SLC − ON image in Flathead Lake, Montana, USA. The rows from top to bottom are the 1, 2, 3, 4, 5, and 7 band images used to train the dictionary and the trained dictionary. For each row from left to right, the first to fifth images are 5 of the 13 images used to train the dictionary, which are displayed in the last column:

(8) $$\begin{array}{c} x=D\alpha \;. \end{array}$$

Among them, *α* ∈ *ℂ*^*M*^ is the coefficient of sparse representation (SR), and its sparsity can be represented by ‖*α*‖_0_. Among them, ‖·‖_0_ is the pseudo-norm of *l*_0_, which is the number of nonzero elements in the coefficient *α*. Substituting the above formula into formula (7), the following formula is obtained:

(9) $$\begin{array}{c} y=\Phi \;D\alpha +\varepsilon ,\\ s.t.\;{\left\|\alpha \right\|}_{0}<k. \end{array}$$

Among them, *k* is the threshold of sparsity constraint.

However, because the coefficient *α* is a non-convex and nondeterministic polynomial difficult optimization problem, it is more difficult to solve the *l*_0_ norm minimization problem of the coefficient *α*. At the same time, when the image contains noise, the solution of the above formula is unstable. To avoid this problem, the convex *l*_1_− norm is used to replace the non-convex *l*_0_− norm; that is, the non-convex optimization problem of the above formula is transformed into the following convex optimization problem for solution:

(10) $$\begin{array}{c} y=\Phi \;D\alpha +\varepsilon \\ s.t.\;{\left\|\alpha \right\|}_{1}<k. \end{array}$$

Algorithms such as alternating direction method (ADM) can effectively optimize the above formula. The above formula can be equivalent to the following unconstrained optimization problem by properly selecting the regularization parameters:

(11) $$\begin{array}{c} \left\{\begin{array}{c} \hat{\alpha }=\underset{\alpha }{\arg\min}{\left\|y-\Phi \;D\alpha \right\|}_{2}^{2}+\lambda {\left\|\alpha \right\|}_{1},\\ \hat{y}=D\hat{\alpha }. \end{array}\right. \end{array}$$

According to the expanded form of the above formula, the structured sparse (SS) image repair model can be realized by the following formula:

(12) $$\begin{array}{c} \left\{\begin{array}{c} \hat{A}=\underset{A}{\arg\min}{\left\|Y-\Phi \;DA\right\|}_{2}^{2}+\lambda {\left\|A\right\|}_{1},\\ \hat{Y}=D\hat{A}. \end{array}\right. \end{array}$$

*Y* is the Landsat − 7ETM + SLC − OFF image. Matrix *A* is the sparse coefficient matrix, $\hat{A}$ is the estimated sparse coefficient matrix, and $\hat{Y}$ is the restored image. Algorithms such as alternate direction method of multipliers (ADMM) and split Bregman can effectively minimize the above formula. In image restoration theory based on structural sparse representation, nonlocal self-similar methods are often used, such as the nonlocal method of Dong et al. [16] and the simultaneous sparse coding of Banerjee and Chatterjee [17] (SSC) method.

The article "Online Education Classroom Intelligent Management System Based on Tensor CS Reconstruction Model" was published in 2022. Journal: Comput Intell Neurosci.

## 5. Image Restoration Algorithm Based on Nonlocal Low-Rank Regularization

For Landsat − 7ETM+SLC − OFF images, a non-convex nonlocal low-rank regularization model is proposed. The non-convex regularization model contains a set of self-similar feature blocks and a low-rank approximation of sparse representation. Nonlocal self-similarity is to intercept a window in the image and select a small image block as a sample image in the window. The sample image block is compared with other image blocks in the window, and *m* − 1 most similar sample image blocks are found, so that there are *m* very similar image blocks in the entire window. Sample image patches and *m* − 1 similar image patches are converted into column vectors, and all column vectors are arranged into a matrix, and then, the rank of this matrix is very low. The low rank of the matrix is very important prior information, which is of great significance to the establishment and solution of the image restoration model.

Since the US Landsat − 7ETM+ image data are a large data set, there are a sufficient number of similar image patches of size $\sqrt{n}\times \sqrt{n}$ in the image *x*, and the given sample image patches *x*_*i*_^\Ω^ are grouped according to similarity. Among them, \Ω represents the effective part; that is, the value of the missing pixel in the vector *x*_*i*_ is set to 0, and the rest of the set of nonzero elements is denoted as *x*_*i*_^\Ω^. The effective part of the image patch does not need to be updated in the image patch repair. A given sample image small block should contain no more than 3-pixel missing data. Among them, the missing pixel value is set to 0.

(13) $$\begin{array}{c} x_{i}^{\backslash \Omega }=R_{i_{j}x}. \end{array}$$

In the image window *x*, small image blocks are intercepted. If the pixel data corresponding to the effective part of the sample image small block are found to be similar to the effective part of the sample image small block at position *j*, then the similar image small block is represented by *x*_*i*_*j*__^\Ω^ ∈ *ℂ*^*n*^. The pixel data in the position of the non-corresponding effective part in the image small block still have the pixel value set to 0. For each sample image small block *x*_*i*_^\Ω^ in a local window, for example, in 70 × 70 or 90 × 90, the *K*-nearest neighbor (KNN) algorithm is used for preliminary classification, as shown in the following formula:

(14) $$\begin{array}{c} G_{i}=\left\{i_{j}|\left\|x_{i}^{\backslash \Omega }-x_{i_{j}}^{\backslash \Omega }\right\|<T\right\}. \end{array}$$

Among them, *T* is the similarity threshold, and *G*_*i*_ is the position of the image patch similar to the sample image patch *x*_*i*_^\Ω^. For there are multiple image patches similar to the sample image patches, only the *m* − 1 most similar image patches are selected. Therefore, we obtain a matrix.

(15) $$\begin{array}{c} x_{i}^{\backslash \Omega }=\left[x_{i_{0}}^{\backslash \Omega },x_{i_{1}}^{\backslash \Omega },\ldots ,x_{i_{m-1}}^{\backslash \Omega }\right],\\ x_{i}^{\backslash \Omega }\in {\mathbb{C}}^{n\times m}. \end{array}$$

Among them, it includes *H* and *m* − 1 most similar patches of the sample image. Among them, *x*_*i*_^\Ω^ is the effective part of the matrix *X*_*i*_, *X*_*i*_ ∈ *ℂ*^*n*×*m*^. It is easy to find that each column of *x*_*i*_^\Ω^ represents a small image block, which is similar to the sample image small block *x*_*i*_^\Ω^. Since the amount of data of Landsat − 7ETM+ image may be too large, for the efficient operation of the subsequent singular value decomposition (SVD) method, the matrix *x*_*i*_^\Ω^ needs to be composed of low rank; that is, several adjacent image patches of the local window are very similar. Therefore, the following similarity discrimination method is established:

(16) $$\begin{array}{c} H_{i}=\left\{\left(i,j\right)|\left\|x_{i}^{\backslash \Omega }-x_{j}^{\backslash \Omega }\right\|<T_{1}\right\}. \end{array}$$

Among them, *T*_1_ is the similarity threshold, and *H*_*i*_ is the position of two similar sample patches. After regrouping, similar image patches are formed using the following method; that is, if the following formula is satisfied, two image patches can also be defined as similar:

(17) $$\begin{array}{c} K_{i,j}=\left\{\left(i,j\right)|\left\|x_{i}^{\backslash \Omega }-x_{j}^{\backslash \Omega }\right\|<\frac{T}{2}\right\},\\ \left\|x_{i}^{\backslash \Omega }-x_{i_{j}}^{\backslash \Omega }\right\|<\frac{T}{2},\\ \left\|x_{i}^{\backslash \Omega }-{\hat{x}}_{j_{k}}^{\backslash \Omega }\right\|<\frac{T}{2}. \end{array}$$

Among them, *x*_*i*_*j*__^\Ω^ and ${\hat{x}}_{j_{k}}^{\backslash \Omega }$ are image patches in *X*_*i*_ and *X*_*j*_, respectively. At the same time, similar image patches meeting the following conditions are searched:

(18) $$\begin{array}{c} M_{i}=\left\{i_{j}|\left\|x_{i}^{\backslash \Omega }-{\hat{x}}_{i_{j}}^{\backslash \Omega }\right\|+\left\|x_{i}^{\backslash \Omega }-{\hat{x}}_{i_{j}}^{\backslash \Omega }\right\|<T\right\}. \end{array}$$

Among all image patches that meet the above conditions, only the most similar *m* patches are selected. If there is no small image block that meets the above conditions, the matrix is not merged. After regrouping the image patches, the merged matrix of the two sample image patches *x*_*i*_^\Ω^ and *x*_*j*_^\Ω^ is obtained:

(19) $$\begin{array}{c} Y_{i}^{\backslash \Omega }=\left[x_{i}^{\backslash \Omega },x_{i_{1}}^{\backslash \Omega },\ldots ,x_{i_{t}}^{\backslash \Omega },x_{j}^{\backslash \Omega },x_{j_{t+1}}^{\backslash \Omega },\ldots ,x_{j_{m-1}}^{\backslash \Omega }\right]. \end{array}$$

Among them, there is *Y*_*i*_ ∈ *ℂ*^*n*×*m*^, and this process is repeated until all small image blocks that satisfy the above formula are merged. The merged image blocks have similar structural features, and the matrix *Y*_*i*_ is low rank.

The article "Online Education Classroom Intelligent Management System Based on Tensor CS Reconstruction Model" was published in 2022. Journal: Comput Intell Neurosci.

In actual situations, *Y*_*i*_^\Ω^ may be corrupted by noise, which leads to deviations from the expected low-rank constraint. The method used here is to decompose matrix *Y*_*i*_^\Ω^ into

(20) $$\begin{array}{c} Y_{i}^{\backslash \Omega }=Z_{i}^{\backslash \Omega }+W_{i}^{\backslash \Omega }. \end{array}$$

Among them, *Z*_*i*_^\Ω^ and *W*_*i*_^\Ω^ represent low-rank matrix and Gaussian noise matrix, respectively. Then, by solving the minimization optimization problem of the following formula, the low-rank matrix *Z*_*i*_^\Ω^ can be calculated.

(21) $$\begin{array}{c} Z_{i}^{\backslash \Omega }=\arg\underset{Z_{i}^{\backslash \Omega }}{\min}rank\left(Z_{i}^{\backslash \Omega }\right),\\ s.t.\;{\left\|Y_{i}^{\backslash \Omega }-Z_{i}^{\backslash \Omega }\right\|}_{F}^{2}\leq \sigma_{w}^{2}. \end{array}$$

In the formula, ‖·‖_*F*_^2^ represents the Frobenius norm, and *σ*_*w*_^2^ is the Gaussian noise variance. However, since the minimization in the above equation is a NP − hard problem, this equation cannot be solved directly. To obtain the approximate solution of the above formula, the convex kernel norm ‖·‖_*∗*_ (singular value sum) regularization model is usually used instead of the low-rank minimization problem. Although the convex kernel norm ‖·‖_*∗*_ model is theoretically mature, many references prove that a smooth and not convex low-rank replacement model will produce better denoising results. Recently, a logdet regularized non-convex approximate replacement model was proposed. The comparison between the non-convex replacement function logdet and the kernel norm replacement function under standard conditions shows that when solving the rank minimization problem, the non-convex logdet replacement function model can approximate the low-rank function better than the kernel norm model.

The article "Online Education Classroom Intelligent Management System Based on Tensor CS Reconstruction Model" was published in 2022. Journal: Comput Intell Neurosci.

Generally speaking, matrix *Z*_*i*_^\Ω^ is neither a square matrix nor a positive semi-definite matrix. The above formula can be rewritten as follows:

(22) $$\begin{array}{c} L\left(Z_{i}^{\backslash \Omega },\varepsilon \right)≔\log\;\det\left({\left(Z_{i}^{\backslash \Omega }{\left(Z_{i}^{\backslash \Omega }\right)}^{T}\right)}^{1/2}+\varepsilon I\right)\\ =\log\;\det\left(U\sum^{1/2}U^{-1}+\varepsilon I\right)\\ =\log\;\det\left(\sum^{1/2}+\varepsilon I\right). \end{array}$$

Among them, ∑ is a diagonal matrix, and the diagonal elements of ∑ are the eigenvalues of matrix *Z*_*i*_^\Ω^(*Z*_*i*_^\Ω^)^*T*^. Matrix *Z*_*i*_^\Ω^(*Z*_*i*_^\Ω^)^*T*^ can be decomposed into orthogonal form:

(23) $$\begin{array}{c} Z_{i}^{\backslash \Omega }{\left(Z_{i}^{\backslash \Omega }\right)}^{T}=U\sum U^{-1}. \end{array}$$

Since ∑^1/2^ is a diagonal matrix, its diagonal elements are the singular values of matrix *Z*_*i*_^\Ω^. To solve for *Z*_*i*_^\Ω^, *Z*_*i*_^\Ω^'s logdet model is used. Therefore, a low-rank approximate model can be obtained as follows:

(24) $$\begin{array}{c} Z_{i}^{\backslash \Omega }=\arg\underset{Z_{i}^{\backslash \Omega }}{\min}L\left(Z_{i}^{\backslash \Omega },\varepsilon \right),\\ s.t.\;{\left\|Y_{i}^{\backslash \Omega }-Z_{i}^{\backslash \Omega }\right\|}_{F}^{2}\leq \sigma_{w}^{2}. \end{array}$$

In fact, the minimization problem of the above formula can be equivalent to the following unconstrained optimization problem:

(25) $$\begin{array}{c} Z_{i}^{\backslash \Omega }=\arg\underset{Z_{i}^{\backslash \Omega }}{\min}\left\|Y_{i}^{\backslash \Omega }-Z_{i}^{\backslash \Omega }\right\|V+\lambda L\left(Z_{i}^{\backslash \Omega },\varepsilon \right). \end{array}$$

For each sample image block in the monitoring image, the low-rank matrix *Z*_*i*_^\Ω^ of the approximate matrix *Y*_*i*_^\Ω^ can be obtained by solving the above formula.

## 6. Model Building

As the gateway layer of the entire system, the wireless router is responsible for the identification of mobile devices, the judgment of entering and leaving the classroom, the recording of attendance time, and the transmission of attendance data. The MAC address is used as the unique identifier of each device, which can be associated with the MAC information of the student and the mobile phone, and the student's identity can be confirmed by obtaining the MAC information of the device. In this system, a wireless router installed with OpenWrt system is used to capture the detection request frame sent by the device at the system data link layer, and the MAC information can be parsed according to the frame format. The wireless network structure model of this system is shown in Figure 1.

The article "Online Education Classroom Intelligent Management System Based on Tensor CS Reconstruction Model" was published in 2022. Journal: Comput Intell Neurosci.

The camera module uses Hikvision DS-2CD893PF-E camera. The camera is directly connected to the router, and the camera network is set. The Linux system timer controls the camera to take pictures of the students in the classroom during class time and stores the pictures on the server. The overall structure of the camera module is shown in Figure 2.

The overall server architecture is shown in Figure 3, which is mainly divided into Web server, Linux server, and database. The tomcat server is built on the Web server side, and all data interaction is in the form of a URL interface. The Linux server uses the Ubuntu system, which is mainly used to control the camera snapshot storage. Using the crontab timer, the start and end time of the course are used as the start time of the timer and write timer for camera snapshot storage task. During class time, the timer is started to start to control the camera to take pictures and upload the picture information to the Web server. The Web server accurately cuts out students' classroom pictures by querying the location information of students' mobile phone attendance, generates personal attendance picture information, and stores it in the database. The relational database MySQL is used as the server database to store student information, teacher information, course information, course selection information, attendance information, picture information, etc.

Around the classroom attendance management, router attendance is designed, which mainly records the time when students go to and from get out of class. The generated attendance information is stored in the database, the timer controls the camera to take pictures during class time, and the pictures are stored in the database. The server calculates the student's course conduct scores based on the router's attendance data and crops the camera shots according to the student's mobile phone sign-in location. Moreover, it makes the traditional classroom attendance more streamlined and standardized, and it conducts all-round classroom management. The data processing relationship between each summary is shown in Figure 4 module relationship.

The article "Online Education Classroom Intelligent Management System Based on Tensor CS Reconstruction Model" was published in 2022. Journal: Comput Intell Neurosci.

The main process receives the message, obtains the MAC information, queries the student information table stdinfo in the database, and queries the student ID through the MAC information to confirm the student's identity. After that, the main process uses the structure linked list to store the association information between the MAC information and the student's student ID and the scan status of the student's mobile phone. The main process traverses the scanning status linked list every ten seconds to determine whether the student is in attendance or sign-out status. After meeting the requirements, the attendance or sign-off information is generated, and the information is sent to the server using CURL, and the information is stored by the server in the attendance information table signinfo in the database. The router obtains the mobile phone MAC information and generates the attendance information as shown in Figure 5.

The client function is completed through the management module, the teacher-student interaction module, and the recommendation reminder module. The server-side function is mainly the system administrator's maintenance function of the system, which is completed by the information management module. The specific overall system function module diagram is shown in Figure 6, and the detailed description of each module is as follows: (1) management module: the management module manages the involved user information and user-related information and includes the registration, modification, and maintenance of user information; the designation, modification, and recording of attendance information; the calculation and viewing of score information; and the arrangement, submission, and inspection of job information. (2) Teacher-student interaction module: the teacher-student interaction module is the interaction between students and teachers in the classroom, including teacher teaching behavior and student feedback behavior. (3) Recommendation module: the recommendation module is the recommendation reminder service introduced above, which mainly includes time reminder, location reminder, learning efficiency reminder, and learning material recommendation. (4) Information management module: the information management module mainly refers to the management and maintenance functions of the system management personnel to ensure the stable, safe, and real-time operation of the system. It mainly includes the entry, modification, and deletion of class information, course information, and user information, as well as certain maintenance of the system.

## 7. System Performance Verification

Next, this article analyzes the performance of the model constructed in this article. The model constructed in this study mainly uses image recognition to identify the characteristics of students and make corresponding strategies based on the recognition results. First, this article analyzes the accuracy of student image feature recognition through 96 sets of data. The results are shown in Table 1 and Figure 7.

The article "Online Education Classroom Intelligent Management System Based on Tensor CS Reconstruction Model" was published in 2022. Journal: Comput Intell Neurosci.

It can be seen from the above chart that the model constructed in this study performs well in the accuracy of teaching image recognition. Next, this article scores the model decision effect, and the results are shown in Table 2 and Figure 8.

The experimental results show that the classroom intelligent management system constructed in this study has good decision-making performance.

## 8. Conclusion

This study uses the tensor CS reconstruction model to construct an online education classroom intelligent management system, uses the cosine function to represent the data energy fitting of the traditional active contour model, and proposes a model based on partial image restoration to fit the energy activity contour of the local cosine, which is used for image and composite image segmentation. The model can segment the composite image with uneven intensity and extract the region of interest in the image. The proposed model is compared with the convex model (CVMST) of Mumford-Shah and the threshold model, the local binary fitting model (LBF), and the L0 regularized Mumford-Shah (L0MS) model. The results show that the model has higher efficiency and robustness for the segmentation of noisy images and blurred images, and the calculation time is close to or faster than these advanced models. In addition, this study uses a discrete form to describe the model, which makes it easier to add a regular term to control the segmentation. Finally, this study uses the improved algorithm proposed to segment the image and obtains the three-dimensional visualization results. The experimental results show that the algorithm proposed in this study has a certain teaching effect.

## Figures and Tables

**Figure 1:** Wireless network structure model.

**Figure 2:** Overall structure of the camera module.

**Figure 3:** Server architecture diagram.

**Figure 4:** Module relationship.

**Figure 5:** Router generates attendance information.

**Figure 6:** System function module diagram.

**Figure 7:** Statistical diagram of the accuracy of model image feature recognition.

**Figure 8:** Statistical diagram of scoring of model classroom management decision.

**Table 1:** Accuracy of model image feature recognition.

No.	Accuracy (%)	No.	Accuracy (%)	No.	Accuracy (%)
1	94.7	33	95.5	65	96.4
2	95.3	34	95.4	66	96.8
3	94.1	35	94.3	67	94.5
4	95.7	36	95.8	68	94.3
5	95.8	37	95.5	69	95.6
6	96.4	38	96.8	70	95.4
7	95.6	39	94.6	71	95.2
8	96.4	40	95.9	72	95.6
9	94.0	41	94.9	73	96.1
10	96.2	42	94.8	74	94.0
11	94.7	43	96.1	75	94.3
12	96.8	44	94.9	76	96.7
13	94.3	45	95.9	77	95.3
14	95.8	46	95.7	78	96.2
15	94.3	47	96.8	79	95.2
16	95.7	48	95.0	80	95.5
17	96.4	49	94.8	81	95.9
18	94.1	50	96.3	82	96.0
19	95.5	51	95.0	83	96.2
20	95.6	52	96.5	84	96.2
21	95.8	53	97.0	85	94.4
22	95.0	54	96.9	86	95.9
23	96.5	55	96.8	87	96.8
24	94.8	56	95.1	88	94.7
25	96.7	57	94.1	89	95.4
26	96.4	58	96.4	90	95.0
27	95.3	59	95.4	91	96.7
28	96.4	60	95.6	92	95.6
29	95.4	61	95.6	93	95.2
30	95.0	62	94.2	94	94.6
31	95.0	63	94.7	95	94.7
32	96.7	64	94.5	96	96.1

The article "Online Education Classroom Intelligent Management System Based on Tensor CS Reconstruction Model" was published in 2022. Journal: Comput Intell Neurosci.

**Table 2:** Statistical table of scoring of model classroom management decision.

No.	Score	No.	Score	No.	Score
1	90.4	33	86.1	65	87.4
2	88.6	34	85.2	66	88.6
3	92.5	35	87.7	67	84.7
4	89.7	36	85.9	68	92.7
5	86.7	37	86.5	69	89.0
6	87.3	38	84.2	70	89.8
7	89.0	39	93.0	71	91.9
8	91.2	40	87.4	72	85.0
9	86.5	41	86.3	73	89.7
10	85.7	42	92.5	74	92.9
11	86.2	43	88.6	75	88.2
12	88.1	44	87.5	76	91.2
13	89.9	45	92.9	77	89.8
14	90.2	46	85.4	78	84.6
15	92.1	47	86.5	79	92.9
16	92.0	48	85.6	80	87.7
17	85.4	49	90.4	81	93.0
18	91.0	50	89.5	82	91.4
19	84.3	51	89.5	83	88.4
20	87.0	52	84.3	84	87.0
21	92.0	53	92.3	85	90.4
22	90.1	54	90.0	86	86.9
23	84.0	55	89.6	87	92.4
24	91.6	56	91.5	88	91.1
25	89.6	57	85.3	89	90.5
26	86.0	58	86.9	90	85.2
27	90.8	59	87.2	91	91.8
28	88.2	60	92.3	92	88.9
29	88.0	61	86.7	93	85.4
30	87.8	62	84.0	94	87.2
31	92.6	63	91.1	95	90.3
32	88.3	64	90.5	96	92.7

## Data Availability

The data used to support the findings of this study are available from the corresponding author upon request.
